# Classification of Mental Stress Using CNN-LSTM Algorithms with Electrocardiogram Signals

**DOI:** 10.1155/2021/9951905

**Published:** 2021-06-04

**Authors:** Mingu Kang, Siho Shin, Jaehyo Jung, Youn Tae Kim

**Affiliations:** AI Healthcare Research Center, Department of IT Fusion Technology, Chosun University, 309 Pilmun-daero Dong-gu, Gwangju 61452, Republic of Korea

## Abstract

The mental stress faced by many people in modern society is a factor that causes various chronic diseases, such as depression, cancer, and cardiovascular disease, according to stress accumulation. Therefore, it is very important to regularly manage and monitor a person's stress. In this study, we propose an ensemble algorithm that can accurately determine mental stress states using a modified convolutional neural network (CNN)- long short-term memory (LSTM) architecture. When a person is exposed to stress, a displacement occurs in the electrocardiogram (ECG) signal. It is possible to classify stress signals by analyzing ECG signals and extracting specific parameters. To maximize the performance of the proposed stress classification algorithm, fast Fourier transform (FFT) and spectrograms were applied to preprocess ECG signals and produce signals in both the time and frequency domains to aid the training process. As the performance evaluation benchmarks of the stress classification model, confusion matrices, receiver operating characteristic (ROC) curves, and precision-recall (PR) curves were used, and the accuracy achieved by the proposed model was 98.3%, which is an improvement of 14.7% compared to previous research results. Therefore, our model can help manage the mental health of people exposed to stress. In addition, if combined with various biosignals such as electromyogram (EMG) and photoplethysmography (PPG), it may have the potential for development in various healthcare systems, such as home training, sleep state analysis, and cardiovascular monitoring.

## 1. Introduction

Stress is a mental and physical reaction that a person may feel when they find themselves in a difficult and/or unfamiliar environment or situation. Excessive stress accumulation can cause chronic diseases such as high blood pressure, heart disease, and cancer and, in severe cases, can lead to death [1, 2]. For this reason, stress observation is becoming increasingly important in modern society.

Studies measuring stress by using various biological signals such as electroencephalography (EEG), electromyogram (EMG), oxygen saturation, and pulse waves have been published [3–5]. However, these measurement methods require expensive and bulky systems to acquire data, are complicated and expensive to use, and require signal analysis by experts.

Existing studies using EEG signals have analyzed stress using support vector machines (SVMs), multilayer perceptrons (MLPs), and naïve Bayes (NB) and have obtained accuracies of 75%, 85.20%, and 64.29%, respectively [6–8]. However, because these studies used only 15 EEGs as training data, underfitting can occur. Furthermore, because an EEG produces a 7-channel signal, it involves a complex and time-consuming process to measure stress signals. Previous studies using EMG signals analyzed by SVM achieved an 85% accuracy. However, despite the same action being taken (the characteristic movement of the muscles), the magnitude of the signal amplitude varies from measurement to measurement, and noise in the signal makes it difficult to extract accurate feature points [9].

Studies that classify stress using an electrocardiogram (ECG) have been the most popular because the signal acquisition method is simpler than other methods and a clear waveform is acquired. Two studies achieved 89.21% and 84.4% accuracy using SVM [10, 11], but extracting feature points can be difficult because of noise and the time required to measure multichannel ECG signals and because preprocessing is not always accurate. Two different studies achieved 75% and 89% accuracy by considering the standard deviation of the R-R interval of the heart rate variability (HRV) signal [12, 13]. Accurate stress classification is difficult because it takes more than 5 min to calculate the standard deviation of the R-R interval, and because the difference in parameter values is minimal. Furthermore, because the ECG waveform is not accurate in the frequency domain, it is difficult to extract feature points, making it difficult to directly evaluate or minimize the effect of noise generated by the human body.

In addition, certain research results have exhibited 63.97% and 82.7% accuracy using fuzzy c-means (FCM) clustering and convolutional neural network (CNN) [14, 15]. These studies have difficulty classifying stress signals because the distance between the center point and the data is slight, and the scale of the training data is small, making it easier for the occurrence of underfitting.

Certain earlier study results have exhibited 87.39% and 90.19% accuracy using CNNs and convolutional recurrent neural networks (CRNNs) [16, 17]. In these studies, the hierarchical structure of the stress classifier is complex, and there is a considerable amount of noise; therefore, it is difficult to achieve a high-stress classification accuracy by detecting an incorrect *R* peak value. Models based on long short-term memory (LSTM) achieved 88.13% accuracy [18]. However, owing to the high noise of the ECG signal, it is difficult to calculate the root mean square (RMS) of the R-R interval.

The aforementioned stress signal classification algorithm using the ECG signal has disadvantages such as underfitting, the calculation of a standard deviation for the R-R interval of a long-time HRV signal, and the detection of an incorrect *R* peak value. To overcome these problems, we propose an ensemble model that accurately classifies mental stress by combining CNN and LSTM. The proposed model extracts the *R* − *S*_peak_ feature point using the threshold value, converts it into a spectrogram, and classifies the stress signal using ECG signal analysis.

To improve the stress classification accuracy, batch normalization (BN), flatten layers, and fully connected layers were added. Subsequently, the accuracy of the stress classification model was improved by separately classifying ECG signals in the time domain and frequency domain. Confusion matrices, receiver operating characteristic (ROC) curves, and precision-recall (PR) curves were used to evaluate the performance of the stress classification model. In this study, we proposed an ensemble method to classify the mental stress of the CNN-LSTM model using ECG signals. The data of the ST Change Database and WESAD Database were trained, and more than 98% classification performance was achieved.

## 2. Materials and Methods

### 2.1. Subject

Figure 1 shows the procedure for classifying stress signals. In this study, we used the ST Change Database and WESAD Database, which provide ECG signals that were acquired in different stress environments. The ST Change Database contains ECG data that records physical stress and consists of 28 ECG signals obtained from 15 male subjects [19]. The WESAD database contains 30 ECG signals measured at the wrist and chest obtained from 15 subjects (12 men and 3 women) [20].

### 2.2. Preprocessing and Feature Extraction

Electrocardiography is the most common way to check health status by noninvasively checking the electrical status of the heart. When taking an electrocardiogram, noise is generated by several factors, which greatly reduces ECG classification accuracy [21]. To solve this problem, we used a low-pass filter and confirmed that 90.89% of the noise was eliminated using a low-pass filter with a sampling frequency of 360 Hz and a cutoff frequency of 150 Hz.

Figure 2 shows the extracted *R* − *S*_peak_ values from an ECG signal. By extracting these data under stress and without stress, the ECG can be accurately analyzed [22]. *R*_peak_ and *S*_peak_ were extracted from ECG signals after setting a threshold. *R*_peak_ extracted the pole when the threshold value was greater than 0.2 mV in one period of the signal and extracted the pole when the threshold value was less than −0.54 mV in one period.

In the under-stress state, the heart beats irregularly and quickly, the R-R interval of the ECG signal becomes narrow, and the *R* − *S*_peak_ increases. On the other hand, in the unstressed state, the heart is relatively stable, the R-R interval widens, and the *R* − *S*_peak_ decreases [23]. In each state, the average *R* − *S*_peak_ without stress was found to be 1.47 mV, and under stress, it was 4.25 mV.  Figure 3 shows the conversion of either signal (under stress or without stress) into a spectrogram.

### 2.3. CNN-LSTM Model Design

Figure 4 shows the architecture of the ensemble model proposed in this study. The classification layer consists of 14 levels.

Table 1 lists the structure of the layers comprising the ensemble model. First, 124 × 124 × 3 image sequence data are input to the sequence input layer. Subsequently, the ECG image data are converted into an array form (vertical, horizontal, and channel) using a sequence folding layer and then transferred to the convolution layer.

The reason for using the sequence folding layer is so that the image sequence data can be converted into an array, arranged, and then transferred to the two-dimensional (2D) convolution layer. The first 2D convolution layer contains six filters of size 5 × 5.

Because of calculating the convolution layer using equation (1), the size of the output value is 124 × 124 × 6. Equation (1) represents the calculation process for the convolution layer. When padding and stride are applied, and the size of the input data and filter is given, the output value can be calculated. *H* and *W* are the input data size, *FH* (filter height) and *FW* (filter weight) are filter size, *S* is the stride, *P* is padding, and *OH* (output height) and *OW* (output weight) are output value sizes.

(1) $$\begin{array}{c} \left(OH,OW\right)=\left(\frac{H+2P-FH}{S}+1,\frac{W+2P-FW}{S}+1\right). \end{array}$$

The output data are then connected to the batch normalization layer. After normalizing the size of the output data to 124 × 124 × 6 in the batch normalization layer, it was connected to the max pooling layer. According to equation (2), the size of the output data is determined by dividing the row and column size by the pooling size.

(2) $$\begin{array}{c} \left(ORs,OCs\right)=\left(\frac{H}{P},\frac{W}{P}\right). \end{array}$$

Its output is fed to a batch normalization layer and then to a max pooling layer. The max pooling layer is a 2 × 2 filter with a stride of 2. As a result, the original data are reduced to a size of 62 × 62 × 6. The second 2D convolution layer contains 12 filters of size 3 × 3. As a result, the data are further reduced to a size of 31 × 31 × 12. Normalization is then performed and the data are passed to the LSTM layer. To transfer the size of the output data to the LSTM layer, normalization was performed using a sequence unfolding layer, and feature vectors were obtained using a flattening layer (or flattened layer).

The flattening layer has the advantage of not affecting the parameter by converting the output of the extracted feature map into a 1D array, which allows reconstructing the feature maps as the input to the LSTM [24]. At this time, the input is transmitted through the hidden layer of the LSTM.

A weight value of 800 × 11532 at the input layer is applied to equations (3)–(7), which represents the computational process of the LSTM layer, to extract the feature value. The LSTM layer consists of input gates (*i*_*t*_, *g*_*t*_), forget gates (*f*_*t*_), and output gates (*O*_*t*_). The LSTM layer is composed of an input gate (*i*_*t*_, *g*_*t*_), forgetting gate (*f*_*t*_), and output gate (*O*_*t*_). In each gate, a weight value is multiplied according to an input vector (*x*_*t*_), a hidden state (*h*_*t*−1_), and a cell state (*C*_*t*_) using the sigmoid and Tanh functions, and then a feature value is extracted.

(3) $$\begin{array}{c} i_{t}=\sigma \left(W_{x}x_{t}+W_{hi}h_{t-1}+b_{i}\right), \end{array}$$

(4) $$\begin{array}{c} g_{t}=\tanh\left(W_{xg}x_{t}+W_{hg}h_{t-1}+b_{g}\right), \end{array}$$

(5) $$\begin{array}{c} f_{t}=\sigma \left(W_{xf}x_{t}+W_{hf}h_{t-1}+b_{f}\right), \end{array}$$

(6) $$\begin{array}{c} O_{t}=\sigma \left(W_{xo}x_{t}+W_{ho}h_{t-1}+b_{o}\right), \end{array}$$

(7) $$\begin{array}{c} C_{t}=f_{t}\circ C_{t-1}+i_{t}\circ g_{t}. \end{array}$$

Subsequently, it is applied to equation (8) to pass the feature value calculated at the output gate to the output layer. Equation (8) is the process of extracting a required feature value from several feature values calculated at the output gate. After extracting a feature value from −1 to 1 using the Tanh function, the feature value in the range calculated using the output gate is transferred to the output layer.

(8) $$\begin{array}{c} h_{t}=O_{t}\circ \;\tanh\left(C_{t}\right). \end{array}$$

The feature value extracted from the LSTM layer classifies the image using a fully connected layer of size two and calculates a probability value for the image classified by the softmax layer. Subsequently, image classification is performed using the feature values extracted earlier using the fully connected layer, and the probability value of the classified image is calculated using the softmax layer. Finally, in the classification step, the signal is classified as either under stress or without stress.

Figure 5 shows the components of the convolution 2D layer and LSTM layer to which equations (1)–(8) are applied. Equations (1) and (2) show the calculation process of the convolution 2D layer among the CNN models, and equations (3)–(7) show the process of outputting feature values using the weight values of the input gate, forgetting the gate, and output gate in the LSTM layer. Equation (8) transfers the feature values in the range from the output gate to the output layer.

We used the confusion matrix, receiver operating characteristic (ROC) curve, and precision-recall (PR) curve to evaluate the stress signal classification performance of the proposed ensemble model [25]. The confusion matrix is a matrix that allows one to evaluate how accurately the predicted value is compared to the actual observed value. We used ECG data from the ST Change Database (DB) and the WESAD DB. The total number of data points was 58. However, with such a small amount of data, it is difficult to accurately evaluate the stress signal classification model. Therefore, to improve the accuracy of the classification model and better analyze its performance, the data were doubled by transforming the time domain data to frequency domain data using the fast Fourier transform (FFT), as indicated in Figure 6. After preprocessing, the performance of the ensemble model was evaluated using 58 time domain data and 58 frequency domain data.

## 3. Experimental Results

Table 2 shows the accuracy, sensitivity, specificity, precision, and negative predictive values obtained to evaluate the classification model's performance using formulas (9)–(13) [26–28]. Formula (1) defines accuracy and indicates the probability of accurately classifying all under stress and without stress conditions. In the formula, TP, TN, FP, and FN indicate true positive, true negative, false positive, and false negative, respectively. For the time and frequency domains, the accuracies of the stress classifier were 94.8% and 98.3%, respectively.

(9) $$\begin{array}{c} \text{Accuracy}=\frac{\text{TP}+\text{TN}}{\text{TP}+\text{TN}+\text{FP}+\text{FN}}. \end{array}$$

Sensitivity refers to the proportion of data correctly classified as without stress to all without stress data (actual observed data). In the time and frequency domains, the sensitivities of the stress classifier were 96.4% and 100%, respectively.

(10) $$\begin{array}{c} \text{Sensitivity}=\frac{\text{TP}}{\text{FN}+\text{TP}}. \end{array}$$

Specificity is the proportion of data correctly classified as under stress among all under stress data (actual observed data). In the time and frequency domains, the sensitivities of the stress classifier were 96.4% and 100%, respectively.

(11) $$\begin{array}{c} \text{Specificity}=\frac{\text{TN}}{\text{TN}+\text{FP}}. \end{array}$$

Precision is the ratio of the data correctly classified by the stress classification algorithm as without stress to the value of all data classified as without stress. In the time and frequency domains, the precision of the stress classifier was 93.1% and 96.6%, respectively.

(12) $$\begin{array}{c} \text{Precision}=\frac{\text{TP}}{\text{TP}+\text{FP}}. \end{array}$$

The negative predictive value is the ratio of data classified correctly as under stress to the actual value without stress data. In the time and frequency domains, the negative predictive values of the stress classifier were 96.6% and 100%, respectively.

(13) $$\begin{array}{c} \text{Negative Predictive Value}=\frac{\text{TN}}{\text{TN}+\text{FN}}. \end{array}$$

Figure 6 shows the results of the classification model's performance using a confusion matrix. The matrix on the left of Figure 7 uses the data converted to the time domain, and the matrix on the right is the result of using the data in the frequency domain. The highest classification accuracy of the proposed ensemble model was 98.3% for the frequency domain. In previous studies, the accuracy of the model was 83.6% [29]. These results indicate that accuracy was improved by 14.7% using the proposed ensemble compared to previous results.

Figure 8 shows the classification performance according to the epochs for the time and frequency domains. The graph shows the mean squared error (MSE) according to the number of epochs. The time domain yielded the lowest MSE at 219 epochs (the validation curve shown), while the frequency domain yielded the lowest MSE at 223 epochs.

Figure 9 shows the ROC curves according to the epochs for the time and frequency domains of the ECG data. The ROC curve is a performance evaluation technique applicable to a binary classifier system that indicates how the performance of the classification model changes as the threshold changes [30]. The area under the curve (AUC) (the area under the ROC curve) is an index used to evaluate the classification performance of different types of signals (stress signals in this study). When the AUC range falls between 0.9 and 1.0 (90%–100%), the classification performance is excellent, and when the AUC range falls between 0.8 and 0.9 (80%–90%), the classifier's performance is low. In the time domain, the AUC of the ROC curve was 94.67%, and it was 98.12% in the frequency domain. The AUC of a previous study was 85.7% [14], and it was confirmed that the ensemble proposed in this study represents a 12.42% improvement. The AUC value of the frequency domain was 3.45% higher than that of the time domain in our model indicating that the classification performance of the stress signal is better in the former.

Figure 10 shows the PR curves for the ECG data according to the epochs for the time and frequency domains. When considering the ROC curve, if the dataset is unbalanced, the shape of the curve is skewed to one side, and the classifier performance cannot be accurately evaluated [31]. The PR curve can be used to overcome the shortcomings of the ROC curve and shows the correlation between precision and recall. The average precision (AP) of the PR curve is an index that can be used to evaluate the classification performance of stress signals [32].

The *X*-axis represents the recall, and the *Y*-axis represents the precision. In the PR curve, the larger the AP is, the better the stress signal classification performance. The PR curve AP of the time domain was 93.8%, and it was 97.6% for the frequency domain. The AP obtained using the PR curve in [32] was 84.2%. Therefore, compared to the previously proposed stress signal classifier, the AP of the PR curve is improved by 13.4% using the proposed classifier. In addition, the AP value of the frequency domain was 3.8% higher than that of the time domain in our model, indicating that the stress classification performance is better in the former.

In previous studies using the time domain or frequency domain of ECG data, the epochs were set to 10, and the batch size was set to 64. As a result, the time domain and frequency domain accuracies were 83.6% and 74.5%, respectively [33]. However, the architectures used are susceptible to overfitting, and the accuracies achieved after 10 epochs may reflect this problem.  Figure 11 shows the accuracy of stress classification using the proposed CNN-LSTM. After setting the epochs to 20 and the batch size to 64, the classification accuracies involving ECG stress signals in the time and frequency domains were measured. Under these settings, the time required for the time domain classification was 7 min 48 s and the verification accuracy was 94.13%. The elapsed time for the frequency domain was 7 min 31 s and the verification accuracy was 98.26%, which represents 10.53% and 23.76% improvements in accuracy compared to previous results [33].

For comparison purposes, we evaluated the stress classification performance of the CNN, LSTM, and CNN-LSTM models. First, stress signals were classified using CNN. After inputting the time series data values from the DBs into the image input layer, feature maps were extracted using convolutional, batch normalization, and max pooling layers. The stress was classified using a fully connected layer and a softmax layer under stress and without stress as the final classification. The classification accuracy of the stress signals using CNN was 88.35%.

In addition, stress signals were classified using LSTM. LSTM is a type of recurrent neural network (RNN), which is an artificial neural network that recognizes patterns in data that can be represented as an array and is used for tasks such as text and gene signal analysis. After inputting the sequence data of the ECG DBs into the sequence input layer, the output was calculated using the LSTM layer (with the ReLU activation function). The signal was then classified as under stress or without stress using a fully connected layer. The classification accuracy of the stress signals using LSTM was 86.25%.

Table 3 compares the stress classification accuracies of the CNN, LSTM, and CNN-LSTM models. We set the epochs to 20 and the batch size to 64 and then determined the elapsed time and accuracy. The results confirmed that the CNN-LSTM model was approximately 1 min faster than the CNN and LSTM models, and accuracy was improved by 9.91% and 12.01%, respectively.

Figure 12 shows the AUC and AP curves for each model based on the ROC and PR results. The AUC of CNN-LSTM was 98.12%, while those of CNN and LSTM were 87.5% and 84.3%, respectively. Therefore, the AUC of the CNN-LSTM model was 10.62% and 13.82% higher than that of the CNN and LSTM models, respectively, confirming that its stress classification performance is better. The AP of CNN-LSTM was 97.6%, and it was 88.2% and 86.02%, respectively, for CNN and LSTM. The CNN-LSTM model achieved AP values that were 9.4% and 11.58% higher than the CNN and LSTM models, respectively, further confirming improved classification performance.

## 4. Discussion

In this study, to improve the performance of stress classification and prevent overfitting, an optimized ensemble model was developed by generating additional data using spectrograms and adding layers such as batch normalization, a flattening layer, and a fully connected layer. The performance of the classifier was evaluated using a confusion matrix, ROC, and other measures. By applying the average value of the *R* − *S*_peak_ of the ECG signal, the characteristics of under-stress and without-stress signals are extracted to improve the stress classification accuracy. In the time domain, a precision of 93.1%, a sensitivity of 96.4%, and a specificity of 93.3% were achieved. In the frequency domain, a precision of 96.6%, a sensitivity of 100%, and a specificity of 96.7% were achieved. The CNN-LSTM achieved 94.8% accuracy for time domain signals and 98.3% accuracy for frequency domain signals. The best stress classification accuracy of the proposed CNN-LSTM algorithm is 98.3%, which is approximately 14.7% higher than the best accuracies reported in previous studies. The proposed stress classifier achieves optimal stress signal classification performance when the number of epochs is 219 in the time domain and 223 in the frequency domain. In addition, the model's performance was evaluated using ROC and PR curves. It was confirmed that improvements of 12.42% and 13.4%, respectively, were obtained compared to previous study results.

## 5. Conclusions

In this study, we proposed an improved ensemble model based on CNN-LSTM to accurately classify stress states. To prevent the overfitting of the algorithm and improve the accuracy of the classifier, ECG signals were classified separately in the time domain and frequency domain. The proposed ensemble model achieved a stress classification accuracy of 98.3%. These results exhibit an approximate 14.7% improvement in accuracy compared to earlier studies that classify the existing under stress and without stress. In the future, we plan to improve the preprocessing method, such as a subtle noise removal of biological signals, and to improve accuracy by applying a wearable transform filter that will remove baseline fluctuations and noise using Fourier transforms. The stress classifier proposed by us is expected to be helpful in mental health management as it can quickly and accurately classify the stress experienced by modern people. It is also expected to assist in preventing various diseases such as depression, high blood pressure, and diabetes through periodic stress management.

## Figures and Tables

**Figure 1:** Procedure for classifying stress signals and validating the model.

**Figure 2:** Feature point extraction by threshold.

**Figure 3:** (a) Without stress ECG converted to a spectrogram. (b) Under stress ECG converted to a spectrogram.

**Figure 4:** Classification architecture.

**Figure 5:** Components of the convolution 2D layer and the LSTM layer.

**Figure 6:** FFT transformation to increase input data quantity.

**Figure 7:** Classification performance evaluation of stress signals using a confusion matrix.

**Figure 8:** Classifier performance evaluation according to epoch.

**Figure 9:** Stress classification performance evaluation using ROC curves.

**Figure 10:** Evaluation of classification performance using PR curve.

**Figure 11:** Time and frequency domain stress signal classification.

**Figure 12:** Evaluation of classification performance of stress signals using ROC and PR curves.

**Table 1:** Classification layers used to evaluate stress signals using CNN-LSTM.

Number	Layer	Activation	Weights	Bias
1	Sequence input layer	124 × 124 × 3	—	—
2	Sequence folding layer	124 × 124 × 1	—	—
3	Convolution 2D layer	124 × 124 × 6	5 × 5 × 3 × 6	1 × 1 × 6
4	Batch normalization layer	124 × 124 × 6	—	—
5	Max pooling layer	62 × 62 × 6	—	—
6	Convolution 2D layer	62 × 62 × 12	3 × 3 × 6 × 12	1 × 1 × 12
7	Batch normalization layer	62 × 62 × 12	—	—
8	Max pooling layer	31 × 31 × 12	—	—
9	Sequence unfolding layer	31 × 31 × 12	—	—
10	Flatten layer	11532	—	—
11	LSTM layer	200	Input: 800 × 11532 recurrent: 800 × 200	800 × 1
12	Fully connected layer	2	2 × 200	2 × 1
13	Softmax layer	2	—	—
14	Classification	—	—	—

**Table 2:** Classification performance assessment of stress signals in time and frequency domains.

Time domain					
Stress	Precision	Sensitivity	Specificity	Negative predictive value	Accuracy

Performance (%)	93.1%	96.4%	93.3%	96.6%	94.8%
Error (%)	6.9%	3.6%	6.7%	3.4%	5.2%

Frequency domain					
Stress	Precision	Sensitivity	Specificity	Negative predictive value	Accuracy

Performance (%)	96.6%	100%	96.7%	100%	98.3%
Error (%)	3.4%	0.0%	3.3%	0.0%	1.7%

**Table 3:** Classification accuracy comparison of stress signals using CNN, LSTM, and CNN-LSTM.

	CNN	LSTM	CNN-LSTM
Elapsed time	8 min 32 s	8 min 45 s	7 min 31 s
Accuracy	88.35%	86.25%	98.26%

## Data Availability

The data are available at https://physionet.org/content/stdb/1.0.0/, https://archive.ics.uci.edu/ml/datasets/WESAD+%28Wearable+Stress+and+Affect+Detection%29.
